# Associations of tumor necrosis factor-α polymorphisms with the risk of colorectal cancer: a meta-analysis

**DOI:** 10.1042/BSR20181750

**Published:** 2019-01-11

**Authors:** Xue Huang, Shanyu Qin, Yongru Liu, Lin Tao, Haixing Jiang

**Affiliations:** Department of Gastroenterology, The First Affiliated Hospital of Guangxi Medical University, Nanning, Guangxi, China

**Keywords:** Colorectal cancer (CRC), Gene polymorphisms, Meta-analysis, Tumor necrosis factor-α (TNF-α)

## Abstract

**Background:** Recently, the roles of tumor necrosis factor-α (*TNF-α*) polymorphisms in colorectal cancer (CRC) were analyzed by some pilot studies, with inconsistent results. Therefore, we performed the present study to better assess the relationship between *TNF-α* polymorphisms and the risk of CRC.

**Methods:** Eligible studies were searched in PubMed, Medline, Embase and CNKI. Odds ratios (ORs) and 95% confidence intervals (CIs) were used to assess correlations between *TNF-α* polymorphisms and CRC.

**Results:** A total of 22 studies were included for analyses. A significant association with the risk of CRC was detected for *TNF-α* -308 G/A (recessive model: *P* = 0.004, OR = 1.42, 95%CI 1.12–1.79) polymorphism in overall analyses. Further subgroup analyses based on ethnicity of participants revealed that *TNF-α* -238 G/A was significantly correlated with the risk of CRC in Caucasians (dominant model: *P* = 0.01, OR = 0.47, 95%CI 0.26–0.86; overdominant model: *P* = 0.01, OR = 2.27, 95%CI 1.20–4.30; allele model: *P* = 0.02, OR = 0.51, 95%CI 0.29–0.90), while -308 G/A polymorphism was significantly correlated with the risk of CRC in Asians (recessive model: *P* = 0.001, OR = 2.23, 95%CI 1.38–3.63).

**Conclusions:** Our findings indicated that *TNF-α* -238 G/A polymorphism may serve as a potential biological marker for CRC in Caucasians, and *TNF-α* -308 G/A polymorphism may serve as a potential biological marker for CRC in Asians.

## Introduction

Colorectal cancer (CRC) refers to malignancy that occurs in the colon and rectum. It is the third most commonly seen cancer in men, and the second commonly seen cancer in women [1]. Despite rapid advances in early diagnosis and surgical treatment over the past few decades, CRC still accounts for approximately one-tenth of cancer-related deaths, making it one of the major threats to public health worldwide [2]. To date, the exact cause of CRC remains unclear. Although smoking, excessive alcohol intake and high consumption of red meat were already identified as potential risk factors of CRC [3–5]. The fact that a significant portion of CRC patients did not expose to any of these carcinogenic factors suggests that genetic susceptibility may play a crucial part in the pathogenesis of CRC [6].

Tumor necrosis factor-α (TNF-α) plays a central role in the regulation of anti-tumor immune responses. Previous clinical investigations showed that serum TNF-α levels in CRC patients were significantly elevated [7], and patients with lower TNF-α levels had better prognosis compared with these with higher TNF-α levels [8,9]. Consequently, functional *TNF-α* polymorphisms were thought to be ideal candidate genetic markers of CRC. Recently, some pilot studies were conducted to investigate associations between *TNF-α* polymorphisms and the risk of CRC. But the results of these studies were conflicting [10–31]. Therefore, we conducted this meta-analysis to better analyze the roles of *TNF-α* polymorphisms in the development of CRC.

## Materials and methods

### Literature search and inclusion criteria

This meta-analysis was performed according to the Preferred Reporting Items for Systematic Reviews and Meta-analyses (PRISMA) guideline [32]. Potentially eligible articles were searched in PubMed, Medline, Embase and CNKI using the combination of following key words: ‘tumor necrosis factor-α’, ‘TNF-α’, ‘polymorphism’, ‘variant’, ‘mutation’, ‘genotype’, ‘allele’, ‘colorectal’, ‘colon’, ‘rectal’, ‘cancer’, ‘tumor’, ‘carcinoma’, ‘neoplasm’ and ‘malignancy’. The initial literature search was conducted in 2018 February and the latest update was performed in 2018 July. The reference lists of all retrieved publications were also screened to identify other potentially relevant articles.

Included studies should meet all the following criteria: (1) case–control study on correlations between *TNF-α* polymorphisms and the risk of CRC; (2) provide adequate data to calculate odds ratios (ORs) and 95% confidence intervals (CIs); (3) full text available. Studies were excluded if one of the following criteria was fulfilled: (1) not relevant to *TNF-α* polymorphisms and CRC; (2) family-based association studies; (3) case reports or case series; (4) abstracts, reviews, comments, letters and conference presentations. For duplicate reports, only the study with the largest sample size was included. No language restrictions were imposed in this meta-analysis.

### Data extraction and quality assessment

The following data were extracted from included studies: (1) name of the first author; (2) year of publication; (3) country and ethnicity of participants; (4) the number of cases and controls and (5) genotypic distributions of *TNF-α* polymorphisms in cases and controls. Additionally, the probability value (*P* value) of Hardy–Weinberg equilibrium (HWE) test was also calculated based on genotypic frequency of *TNF-α* polymorphisms in the control group.

The Newcastle–Ottawa scale (NOS) was employed to assess the quality of eligible studies from three aspects: (1) selection of cases and controls; (2) comparability between cases and controls and (3) exposure in cases and controls [33]. The NOS has a score range of zero to nine, and studies with a score of more than seven were thought to be of high quality.

Two reviewers (Huang and Qin) conducted data extraction and quality assessment independently. When necessary, the reviewers wrote to the corresponding authors for extra information or raw data. Any disagreement between two reviewers was solved by discussion with the third reviewer (Jiang) until a consensus was reached.

### Statistical analyses

All statistical analyses in the present study were conducted with Review Manager Version 5.3.3 (The Cochrane Collaboration, Software Update, Oxford, United Kingdom). ORs and 95% CIs were used to assess potential associations of *TNF-α* polymorphisms with the risk of CRC in the dominant, recessive, overdominant and allele models, and a *P* value of 0.05 or less was considered to be statistically significant. Between-study heterogeneity was evaluated based on *Q* test and *I*^2^ statistic. If *P* value of *Q* test was less than 0.1 or *I*^2^ was greater than 50%, random-effect models (REMs) would be used for analyses due to the existence of significant heterogeneities. Otherwise, fixed-effect models (FEMs) would be applied for analyses. Subgroup analyses by ethnicity of participants were subsequently conducted to obtain more specific results. Sensitivity analyses were carried out to test the stability of the results. Funnel plots were applied to evaluate possible publication bias.

## Results

### Characteristics of included studies

The literature search identified 389 potentially relevant articles. After exclusion of irrelevant and duplicate articles by reading titles and abstracts, 42 articles were retrieved for further evaluation. Another 20 articles were subsequently excluded after reading the full text. Finally, a total of 22 eligible studies were included in this meta-analysis (see Figure 1). Characteristics of included studies were summarized in Table 1.

**Figure 1:** Flowchart of study selection for the present study

**Table 1:** The characteristics of included studies for *TNF-α* polymorphisms and CRC

First author, year	Country	Ethnicity	Source of controls	Sample size	Genotype distribution		*P*-value for HWE	NOS score
					Cases	Controls		
**-238 G/A**					GG/GA/AA			
Garrity-Park 2008 [13]	USA	Mixed	HB	114/114	109/5/0	107/6/1	0.017	8
Gutiérrez-Hurtado 2016 [15]	Mexico	Mixed	PB	143/49	127/14/2	42/6/1	0.199	7
Hamadien 2016 [16]	Saudi Arabia	Caucasian	PB	100/100	86/13/1	97/2/1	<0.001	8
Jang 2001 [17]	Korea	Asian	PB	27/92	27/0/0	80/11/1	0.391	8
Kapitanović 2014 [18]	Croatia	Caucasian	PB	200/200	181/18/1	188/11/1	0.076	8
Madani 2008 [24]	Iran	Caucasian	PB	51/46	51/0/0	45/1/0	0.941	7
Wang 2008 [31]	China	Asian	PB	343/670	320/22/1	620/50/0	0.316	8
**-308 G/A**					GG/GA/AA			
Banday 2016 [10]	India	Caucasian	PB	142/184	124/18/0	150/34/0	0.167	8
Basavaraju 2015 [11]	UK	Caucasian	PB	388/495	253/117/18	309/167/19	0.543	7
Burada 2013 [12]	Romania	Caucasian	PB	144/233	115/26/3	189/42/2	0.842	8
Garrity-Park 2008 [13]	USA	Mixed	HB	114/114	52/49/13	92/20/2	0.464	8
Gunter 2006 [14]	USA	Mixed	PB	217/202	146/59/12	139/57/6	0.957	8
Gutiérrez-Hurtado 2016 [15]	Mexico	Mixed	PB	164/209	139/21/4	180/27/2	0.392	7
Hamadien 2016 [16]	Saudi Arabia	Caucasian	PB	100/100	67/23/10	59/23/18	<0.001	8
Jang 2001 [17]	Korea	Asian	PB	27/92	24/3/0	85/7/0	0.704	8
Kapitanović 2014 [18]	Croatia	Caucasian	PB	200/200	163/35/2	163/35/2	0.937	8
Landi 2003 [19]	France	Caucasian	PB	363/320	278/80/5	234/76/10	0.220	7
Li 2011 [21]	China	Asian	PB	180/180	156/15/9	160/19/1	0.599	8
Li 2017 [22]	China	Asian	PB	569/570	500/66/3	493/75/2	0.632	8
Macarthur 2005 [23]	UK	Caucasian	PB	246/389	157/74/15	224/145/20	0.577	8
Park 1998 [25]	Korea	Asian	PB	136/331	40/71/25	148/151/32	0.465	7
Stanilov 2014 [26]	Bulgaria	Caucasian	PB	119/177	88/28/3	135/40/2	0.612	8
Suchy 2008 [27]	Poland	Caucasian	PB	350/350	254/87/9	248/95/7	0.546	8
Theodoropoulos 2006 [28]	Greece	Caucasian	PB	222/200	152/56/14	146/44/10	0.010	7
Toth 2007 [29]	Hungary	Caucasian	PB	183/141	132/48/3	111/30/0	0.157	7
Tsilidis 2009 [30]	USA	Mixed	PB	204/372	146/55/3	275/90/7	0.908	7
Wang 2008 [31]	China	Asian	PB	344/669	284/58/2	554/111/4	0.538	8
**-857 C/T**					CC/CT/TT			
Garrity-Park 2008 [13]	USA	Mixed	HB	114/114	98/16/0	92/22/0	0.254	8
Hamadien 2016 [16]	Saudi Arabia	Caucasian	PB	100/100	85/15/0	85/15/0	0.417	8
Kapitanović 2014 [18]	Croatia	Caucasian	PB	200/200	130/64/6	126/67/7	0.599	8
Landi 2006 [20]	Spain	Caucasian	PB	281/268	219/58/4	220/45/3	0.684	7
Suchy 2008 [27]	Poland	Caucasian	PB	350/350	253/88/9	242/98/10	0.983	8
**-863 C/A**					CC/CA/AA			
Garrity-Park 2008 [13]	USA	Mixed	HB	114/114	84/28/2	80/33/1	0.224	8
Suchy 2008 [27]	Poland	Caucasian	PB	350/350	262/77/11	257/83/10	0.302	8
**-1031 T/C**					TT/TC/CC			
Garrity-Park 2008 [13]	USA	Mixed	HB	114/114	79/31/4	75/36/3	0.588	8
Kapitanović 2014 [18]	Croatia	Caucasian	PB	200/200	132/56/12	135/54/11	0.082	8
Suchy 2008 [27]	Poland	Caucasian	PB	350/350	250/90/10	227/107/16	0.460	8

Abbreviations: CRC, colorectal cancer; HWE, Hardy–Weinberg equilibrium; NA, not available; NOS, Newcastle–Ottawa scale; TNF-α, tumor necrosis factor-α.

### Overall and subgroup analyses

To investigate potential correlations of *TNF-α* polymorphisms with the risk of CRC, 7 studies about *TNF-α* -238 G/A polymorphism (901 cases and 1179 controls), 20 studies about *TNF-α* -308 G/A polymorphism (4412 cases and 5528 controls), 5 studies about *TNF-α* -857 C/T polymorphism (1045 cases and 1032 controls), 2 studies about *TNF-α* -863 C/A polymorphism (464 cases and 464 controls) and 3 studies about *TNF-α* -1031 T/C polymorphism (664 cases and 664 controls) were enrolled for analyses. A significant association with the risk of CRC was detected for *TNF-α* -308 G/A (recessive model: *P* = 0.004, OR = 1.42, 95%CI 1.12–1.79) polymorphism in overall analyses.

Further subgroup analyses based on ethnicity of participants revealed that *TNF-α* -238 G/A was significantly correlated with the risk of CRC in Caucasians (dominant model: *P* = 0.01, OR = 0.47, 95%CI 0.26–0.86; overdominant model: *P* = 0.01, OR = 2.27, 95%CI 1.20–4.30; allele model: *P* = 0.02, OR = 0.51, 95%CI 0.29–0.90), while -308 G/A polymorphism was significantly correlated with the risk of CRC in Asians (recessive model: *P* = 0.001, OR = 2.23, 95%CI 1.38–3.63). No any other positive results were found for investigated polymorphisms in overall and subgroup analyses (see Table 2).

**Table 2:** Overall and subgroup analyses for *TNF-α* polymorphisms and CRC

Polymorphisms	Population	Sample size	Dominant comparison		Recessive comparison		Overdominant comparison		Allele comparison	
			*P* value	OR (95%CI)	*P* value	OR (95%CI)	*P* value	OR (95%CI)	*P* value	OR (95%CI)
**-238 G/A**	Overall	901/1179	0.72	0.94 (0.68–1.31)	0.94	1.04 (0.34–3.20)	0.68	1.07 (0.77-1.51)	0.77	0.95 (0.70–1.31)
	Caucasian	351/346	**0.01**	**0.47 (0.26–0.86)**	1.00	1.00 (0.14–7.15)	**0.01**	**2.27 (1.20-4.30)**	**0.02**	**0.51 (0.29–0.90)**
	Asian	370/762	0.31	1.29 (0.79–2.12)	0.34	2.69 (0.35–20.78)	0.26	0.75 (0.45–1.24)	0.38	1.24 (0.77–2.00)
**-308 G/A**	Overall	4412/5528	0.30	0.92 (0.78–1.08)	**0.004**	**1.42 (1.12–1.79)**	0.84	0.99 (0.90–1.09)	0.17	0.90 (0.77–1.05)
	Caucasian	2457/2789	0.21	1.08 (0.96–1.22)	0.76	1.05 (0.77–1.42)	0.15	0.91 (0.80–1.03)	0.32	1.06 (0.95–1.17)
	Asian	4412/5528	0.27	0.83 (0.60–1.15)	**0.001**	**2.23 (1.38–3.63)**	0.90	1.01 (0.83–1.24)	0.16	0.81 (0.60–1.09)
**-857 C/T**	Overall	1045/1032	0.62	1.05 (0.86–1.28)	0.85	0.94 (0.50–1.78)	0.66	0.95 (0.78–1.17)	0.62	1.05 (0.87–1.25)
	Caucasian	931/918	0.85	1.02 (0.83–1.26)	0.85	0.94 (0.50–1.78)	0.89	0.99 (0.80–1.22)	0.82	1.02 (0.85–1.23)
**-863 C/A**	Overall	464/464	0.50	1.11 (0.83–1.48)	0.68	1.19 (0.53–2.68)	0.40	0.88 (0.65–1.19)	0.64	1.06 (0.82–1.38)
**-1031 T/C**	Overall	664/664	0.16	1.18 (0.94–1.48)	0.58	0.86 (0.50–1.47)	0.22	0.86 (0.68–1.09)	0.16	1.15 (0.95–1.40)
	Caucasian	550/550	0.20	1.18 (0.92–1.52)	0.47	0.81 (0.45–1.44)	0.31	0.87 (0.67–1.14)	0.17	1.16 (0.94–1.44)

Abbreviations: CI, confidence interval; CRC, colorectal cancer; NA, not available; OR, odds ratio; TNF-α, tumor necrosis factor-α.

For -238 G/A, Dominant comparison: G/A + A/A vs. G/G; Recessive comparison: A/A vs. G/G + G/A; Overdominant comparison: G/G + A/A vs. G/A; Allele comparison: G vs. A.

For -308 G/A, Dominant comparison: G/A + A/A vs. G/G; Recessive comparison: A/A vs. G/G + G/A; Overdominant comparison: G/G + A/A vs. G/A; Allele comparison: G vs. A.

For -857 C/T, Dominant comparison: C/T + T/T vs. C/C; Recessive comparison: T/T vs. C/C + C/T; Overdominant comparison: C/C + T/T vs. C/T; Allele comparison: C vs. T.

For -863 C/A, Dominant comparison: C/A + A/A vs. C/C; Recessive comparison: A/A vs. C/C + C/A; Overdominant comparison: C/C + A/A vs. C/A; Allele comparison: C vs. A.

For -1031 T/C, Dominant comparison: T/C + C/C vs. T/T; Recessive comparison: C/C vs. T/T + T/C; Overdominant comparison: T/T + C/C vs. T/C; Allele comparison: T vs. C.

### Sensitivity analyses

Sensitivity analyses were carried out to examine the stability of meta-analysis results by eliminating studies that deviated from HWE. No changes of results were observed in any comparisons, which indicated that our findings were statistically reliable.

### Publication biases

Potential publication biases in the current study were evaluated with funnel plots. No obvious asymmetry of funnel plots was observed in any comparisons, which suggested that our findings were unlikely to be influenced by severe publication biases.

## Discussion

To the best of our knowledge, this is so far the most comprehensive meta-analysis on correlations between *TNF-α* polymorphisms and CRC. A significant association with the risk of CRC was detected for *TNF-α* -308 G/A polymorphism in overall analyses. Further subgroup analyses based on ethnicity of participants revealed that *TNF-α* -238 G/A was significantly correlated with the risk of CRC in Caucasians, while -308 G/A polymorphism was significantly correlated with the risk of CRC in Asians. No any other positive results were found for investigated polymorphisms in overall and subgroup analyses. The stability of the synthetic results was subsequently evaluated in sensitivity analyses, and no changes of results were observed in any comparisons, which indicated that our findings were quite stable and reliable.

It is worth noting that -238 G/A and -308 G/A polymorphisms were two functional polymorphisms located in the promoter region of *TNF-α*, and the mutant alleles of these two polymorphisms were both associated with a higher expression level of *TNF-α* [10–15]. Thus, it is rational to speculate that subjects carrying mutant alleles of these two polymorphisms may have a relatively lower risk of CRC. From our results, you can see that the trends of developing CRC for these two polymorphisms in overall population are quite similar. But opposite findings were detected in further subgroup analyses. These contradictory findings in subgroup analyses may partially attribute to quite different genetics distributions of these two polymorphisms in Asians and Caucasians. Another possible explanation of this phenomenon is that genetic associations between *TNF-α* polymorphisms and CRC may also be influenced by gene-gene and gene-environmental interactions, but the extent of impact of gene–gene and gene–environmental interactions on genetic association between *TNF-α* polymorphisms and CRC in different ethnicities may be different.

As for evaluation of heterogeneities, obvious between-study heterogeneities were detected for -308 G/A polymorphisms in certain comparisons (data not shown). In further stratified analyses, a great reduction in heterogeneity was found in the Asian subgroup. However, the reduction tendency of heterogeneity in Caucasians was not obvious. These findings suggested that differences in ethnic background could partially explain observed heterogeneities between studies.

As with all meta-analysis, the present study certainly has some limitations. First, our results were based on unadjusted estimations due to lack of raw data, and failure to perform further stratified analyses according to age, gender and co-morbidity conditions may affect the reliability of our findings [34,35]. Second, only case-control studies were included in this meta-analysis, and thus our findings may also be influenced by potential selection bias [35,36]. Third, associations between *TNF-α* polymorphisms and CRC may also be influenced by gene-gene and gene-environmental interactions. However, the majority of studies did not consider these potential interactions, which impeded us to perform relevant analyses accordingly [37,38]. Taken these limitations into consideration, the results of the current study should be interpreted with caution.

Overall, our meta-analysis suggested that *TNF-α* -238 G/A polymorphism may serve as a potential biological marker for CRC in Caucasians, and *TNF-α* -308 G/A polymorphism may serve as a potential biological marker for CRC in Asians. However, further well-designed studies are warranted to confirm our findings. Additionally, future investigations are needed to explore potential roles of other *TNF-α* polymorphisms in the development of CRC.

## Abbreviations

CI: 95% confidence interval
CRC: colorectal cancer
HWE: Hardy–Weinberg equilibrium
NOS: Newcastle–Ottawa scale
OR: odds ratio
TNF-α: tumor necrosis factor-α
